# Biological Functions of Diallyl Disulfide, a Garlic-Derived Natural Organic Sulfur Compound

**DOI:** 10.1155/2021/5103626

**Published:** 2021-10-29

**Authors:** Xiuxiu Song, Ziqi Yue, Lulingxiao Nie, Pengfei Zhao, Kangjian Zhu, Qi Wang

**Affiliations:** ^1^State Key Laboratory of Oral Diseases, National Clinical Research Center for Oral Diseases, West China Hospital of Stomatology, Sichuan University, Chengdu, China; ^2^Department of Prosthodontics, West China Hospital of Stomatology, Sichuan University, Chengdu, China

## Abstract

Garlic is widely accepted as a functional food and an excellent source of pharmacologically active ingredients. Diallyl disulfide (DADS), a major bioactive component of garlic, has several beneficial biological functions, including anti-inflammatory, antioxidant, antimicrobial, cardiovascular protective, neuroprotective, and anticancer activities. This review systematically evaluated the biological functions of DADS and discussed the underlying molecular mechanisms of these functions. We hope that this review provides guidance and insight into the current literature and enables future research and the development of DADS for intervention and treatment of multiple diseases.

## 1. Introduction

Plants are excellent sources of pharmacologically active ingredients. Garlic has been commonly accepted as a functional food and traditional herb for the prevention and treatment of several diseases, especially cancer and infectious diseases [1–4]. It is believed that organic sulfur compounds are responsible for most of the biological activities of garlic [5]. Diallyl disulfide (DADS; structure: two sulfur atoms with two allyl groups; see Figure 1) is a major organosulfur compound of garlic [6, 7]. Studies have shown that DADS has many biological functions, including anti-inflammatory, antioxidant, anticancer, and detoxifying effects, which may be determined by its chemical structure [4, 7–9]. Previous reviews have discussed the promising value of DADS in the prevention and treatment of a wide range of diseases [6]. In this work, we performed a systematic review of the biological functions of DADS based on the cellular and molecular mechanisms, hoping to provide an updated scientific basis and insight for future experiments.

## 2. Methodologies

We made a search in PubMed, Web of Science, and GeenMedical up to June 2021 for the existing literature on DADS. We also searched the International Clinical Trials Registry Platform and ClinicalTrials.gov for potentially relevant clinical trials. References of included papers and reviews were manually searched to make a supplement.

## 3. Biological Functions of DADS

### 3.1. Anti-Inflammatory Activity

Inflammation is an adaptive response of the host to adverse stimuli such as trauma, toxicity, and microbial infection. A proper inflammatory response can eliminate harmful stimuli and promote tissue healing [10]. However, uncontrolled inflammation leads to sustained damage of the tissues and organs often resulting in pathological changes to these systems [11]. Researchers have reported that DADS can inhibit inflammation in several diseases, such as enteritis, arthritis, and pancreatitis [12–14]. Fasolino et al. [15] demonstrated that edema of the mucosa and submucosa was significantly reduced in the colon of rats treated with DADS. Furthermore, a low dose of DADS (between 0.3 and 10 mg/kg) was observed to suppress increases in the colon weight/colon length ratios that represent dinitrobenzene sulfonate-induced intestinal inflammation/damage. In a recent animal study, the anti-inflammatory and antioxidant effects of DADS were further confirmed using a carrageenan injection-induced acute inflammatory response mouse paw model [9].

DADS plays an essential role in inflammatory response by modulating immune cells. Hashizume et al. [16] reported that DADS could modulate the circulating number of total lymphocytes, leukocytes, and monocytes in both dose- and time-dependent manners. Immune cells usually activate intracellular signaling pathways to respond appropriately to adverse stimuli. One of the most important pathways is the nuclear factor kappa B (NF-*κ*B) signaling pathway. A study showed that DADS attenuated the development of cerulein-induced pancreatitis and its associated lung injury in mice by suppressing the transcriptional activity of NF-*κ*B p65 and the degradation of I*κ*B [14], which were consistent with other study findings [17, 18]. Further research revealed that DADS inhibited glycogen synthase kinase (GSK)-3*β*, which suppressed the NF-*κ*B pathway and further prevented prolonged inflammation, cellular transformation, and tissue damage [19]. DADS affected the expression of signal transducer and activator of transcription 1 (STAT 1), which could inhibit the enhancement of NF-*κ*B signaling by binding to the target of tumor necrosis factor (TNF)-*α* [20]. In addition, DADS was shown to suppress the receptor activator of NF-*κ*B ligand-induced inflammatory osteolysis by inhibiting STAT3 and NF-*κ*B signaling both *in vitro* and *in vivo* [21].

One of the most prominent features of the inflammatory response is the release of inflammatory mediators. One study provided strong evidence that DADS could inhibit the lipopolysaccharide (LPS)-induced production of inducible nitric oxide synthase (iNOS) and cyclooxygenase-2 (Cox-2) in RAW 264.7 cells [22], which thus led to the reduction in NO and prostaglandin E2 (PGE2) in activated cells [23–25]. Another study on LPS-stimulated neurogenic innate immune cells, BV2 microglia, also found that treatment with DADS significantly inhibited several proinflammatory cytokines and chemokines, including interleukin (IL)-1*β*, IL-6, TNF-*α*, and monocyte chemoattractant protein-1 [26]. Recent studies have further confirmed this physiological effect in animal models of neuroinflammation [27].

### 3.2. Antioxidant Activity

Antioxidants are substances that prevent, reduce, or repair tissue damage caused by reactive oxygen species (ROS). Over the past two decades, several studies have shown that DADS has a range of antioxidant properties [9, 28–30]. This includes a direct effect on ROS production, which was identified in an *in vitro* study demonstrating that DADS reduced deoxycholic acid-induced ROS levels in Barrett's epithelial cells when introduced within an effective concentration range [31]. Another study showed that treatment with DADS significantly reduced ROS levels in IL-1*β*-treated bone marrow mesenchymal stem cells [17]. However, Filomeni et al. [32] found that DADS induced oxidative stress in neuroblastoma SH-SY5Y cells, which was consistent with the findings of a study on human lung carcinoma cells [33]. This finding aligned with that of other sulfur-containing compounds from garlic, such as diallyl trisulfide (DATS), which induced the apoptosis of human breast cancer cells through ROS accumulation and inhibited it in high glucose-induced cardiomyocytes by reducing ROS production [34, 35]. The discrepancies in these studies may be attributed to the specificity of the tumor cells and differences in the therapeutic dosage of DADS employed in each study. A study on PC12 neuronal cells found that treatment with 20 *μ*M DADS did not exert any evident effect on cell activity. However, the levels of free radicals and membrane lipid peroxidation increased significantly when these cells were treated with concentrations above 50 *μ*M. In addition, there was an increased risk for cytotoxicity when 100 *μ*M of DADS was administered to these cells [36]. The results of this study were similar to those observed in the neuron cell line, N18D3 [37].

Treatment with DADS can activate antioxidant enzymes, such as glutathione S-transferase (GST), catalase, heme oxygenase-1 (HO-1), and superoxide dismutase, which can convert peroxides into less toxic or harmless substances via oxidation reduction, thereby protecting a wide range of cells and tissues from ROS [30, 38, 39]. Treatment with DADS significantly increased nuclear factor-erythroid-2-related factor 2 (Nrf2) and HO-1 levels in acute ethanol-intoxicated mice, ethanol-induced human normal liver cells [40], and LPS-stimulated RAW264.7 cells [41]. Lee et al. [18] demonstrated that DADS promoted the transcription of antioxidant enzymes by dose-dependently enhancing the stability and nuclear translocation of Nrf2 in the cytoplasm. The effects of DADS on Nrf2 also exerted anti-inflammatory effects by deactivating the redox-sensitive proinflammatory NF-*κ*B pathway [42]. In addition, DADS could restore the reduced catalase activity associated with hydrogen peroxide treatment in intestinal porcine epithelial cells [43].

### 3.3. Antimicrobial Activity

#### 3.3.1. Antibacterial Activity

In recent years, antibiotic resistance has become a major health problem. Garlic is believed to be an alternative or complementary medicine for antibiotics owing to its extensive antibacterial properties [44, 45]. Studies have demonstrated that garlic extracts could weaken the formation of *Pseudomonas aeruginosa* biofilms and sensitize them to tobramycin and phagocytosis by polymorphonuclear leukocytes [46]. According to further research, DADS reduced the production of virulence factors, such as elastase, pyocyanin, and swarming motility, in *Pseudomonas aeruginosa* by blocking the inactivation of quorum-sensing (QS) genes [47–49]. The anti-QS effect of DADS was also found to inhibit *Hafnia alvei* H4 by downregulating the expression of luxI and luxR genes [50]. However, the mechanisms by which QS regulates these functions remain unclear. DADS was reported to prevent methicillin-resistant *Staphylococcus aureus* infection in diabetic mice [51], inhibit the growth of *Escherichia coli* as an adjunct of gentamicin [52, 53], suppress the activity of *Helicobacter pylori* both *in vitro* and *in vivo* [54, 55], and reduce the pathogenicity of common microorganisms isolated from ear infections [56]. In addition, several recent studies have demonstrated that DADS could modulate the gut microbiota. H_2_S gas released after treatment with DADS prevented or reversed the naproxen-induced changes in the composition of the intestinal microbiota [57]. According to an *in vivo* study, when a low dose of DADS was added to the normal diet of mice, the bacterial level of *Bacteroides* in their intestinal tract decreased, while that of *Firmicutes* increased [58].

#### 3.3.2. Antifungal Activity

To evaluate the antifungal effect of DADS, Alam et al. [59] administered DADS to mice infected with *Candida albicans*. They found that the niosomal formulation of DADS markedly decreased the secretion of protease and phospholipase from *Candida albicans* and increased the survival of the infected animals. DADS was also reported to inhibit the growth of *Aspergillus versicolor* and its toxic metabolites [60].

#### 3.3.3. Antiviral Activity

The antiviral effect of DADS was first reported in 1993. In this research, DADS inhibited the proliferation of HIV-1-infected cells [61]. In addition, DADS exerted anti-inflammatory and antioxidant effects in a dengue virus study, reducing the symptoms and severity of the disease [62]. In recent reports, garlic has been recommended as a potential medicine for COVID-19 based on the findings of several preclinical and clinical studies [63, 64]. In the molecular docking test, garlic essential oil also showed a good inhibitory effect on SARS-CoV-2 [65, 66]. However, it is still unclear whether DADS plays a role in the anti-SARS-CoV-2 effect of garlic, and further studies are needed.

### 3.4. Detoxification

Numerous studies have shown that DADS can protect organs from the harmful effects of several chemical compounds [4]. For instance, DADS can reduce the hearing loss caused by aminoglycoside drugs [67], attenuate the side effects of gentamicin and cisplatin [67–69], positively affect carbon-tetrachloride-induced hepatic damage [18, 70], relieve haemorrhagic cystitis induced by cyclophosphamide in rats [71, 72], decrease cyclophosphamide-induced developmental toxicity [73], and greatly alleviate the methotrexate-induced decline in kidney function and subsequent kidney damage [74].

DADS can promote detoxification of the body, which is believed to be related to the activation of antioxidant enzymes and phase II enzymes via the Nrf2/ARE pathway. DADS was found to significantly boost the activities of phase II enzymes, including GST, quinone reductase, microsomal epoxide hydrolase, and UDP-glucuronosyltransferase in the liver, intestine, kidney, and lungs [75, 76]. DADS also upregulated the expression of the pi class of GST through JNK/AP-1 and ERK/AP-1 signaling pathways. GST is known to combine with electrophilic compounds in cells to cause detoxification [77].

It has been reported that DADS primarily suppresses the carcinogenic effects of chemical compounds via two mechanisms: the modulation of cytochrome P450 (CYP)-dependent monooxygenase to inhibit carcinogen activation and the induction of phase II enzymes to accelerate carcinogen degradation. DADS exerted its anticarcinogenic effect by inhibiting CYP2E1 levels in humans, and CYP2A3 and CYP2A3 levels in rats induced by methyl-n-pentylnitrosamine [78]. Based on animal studies, the administration of DADS to rats through gastric intubation reduced the amount of liver CYP2E1 protein by 25% [79]. Furthermore, treatment with DADS was found to induce the activation of phase II enzymes by protecting Nrf2 from proteasomal degradation of Keap1 and promoting Nrf2 nuclear accumulation, thereby inhibiting the occurrence of chemical-induced papilloma in mice [80]. A study showed that DADS inhibited cell proliferation, G2/M arrest, H_2_O_2_ formation, and DNA damage induced by ben-zo[a]pyrene, thereby inhibiting the occurrence of breast cancer [81]. DADS also inhibited the expression of serotonin N-acetyltransferase genes and proteins, leading to the reduction of N-acetyl-2-aminofluorene-DNA adducts, which could reduce the risk of cancer associated with exposure to environmental carcinogens [82, 83].

### 3.5. Cardiovascular Protection

The intake of garlic can effectively reduce the risk factors associated with cardiovascular diseases [3, 84, 85]. Based on existing research, DADS plays a critical role in the cardiovascular protective effect exhibited by garlic, by acting as an angiogenesis inhibitor. Exposure to DADS significantly inhibited the angiogenic differentiation of endothelial cells by reducing the activation of matrix metalloproteinases (MMPs) and the secretion of tissue inhibitor of metalloproteinase-1 in endothelial morphogenesis [86, 87]. DADS was also found to effectively downregulate both the transcription and expression of vascular endothelial growth factors in HL-60 cells in time- and dose-dependent manners [88, 89]. Increasing evidence suggests that both connexins and gap junctions are involved in cardiovascular diseases [90]. DADS was observed to improve rat liver epithelial cell gap-junctional intercellular communication, regulate vascular smooth muscle cell proliferation, and significantly increase connexin 43 expression, which is very important for maintaining normal vascular function [91, 92]. Furthermore, DADS is an effective agent against atherosclerosis as it can protect low-density lipoprotein (LDL) from oxidation and glycation [93, 94]. DADS also protected endothelial cells from oxidized LDL (ox-LDL) damage by reversing the inactivation of endothelial NOS (eNOS) by ox-LDL [95].

DADS induces vasodilation by activating perivascular sensory nerve endings [96]. A recent study found that DADS strongly inhibited angiotensin-converting enzyme, upregulated the expression of prostacyclin and Cox-2 in SVEC4-10 cells, and reduced the level of ROS, thereby playing a role in vasodilation [22]. According to reports, DADS could downregulate intercellular adhesion molecule-1 and MMP-9 and block the inactivation of eNOS [95, 97], which has been demonstrated to relieve pulmonary hypertension [98]. Of note, impaired endogenous H_2_S production may be one of the mechanisms underlying hypertension. As DADS is an H_2_S-releasing agent, it could be considered a promising drug for the treatment of cardiovascular disease [99].

Various studies have suggested that DADS protects the heart, and treatment with DADS was found to improve cardiac dysfunction by inhibiting death receptor-dependent and mitochondrial-dependent apoptotic pathways and enhancing the PI3K/Akt pathway in diabetic rats [100]. Furthermore, DADS ameliorated myocardial hypertrophy by enhancing the biogenesis and biological function of mitochondria in the rat heart [101]. The mitochondrial lipid peroxidation product, tans-crotonaldehyde, is known to cause myocardial ischemia by damaging mitochondrial genes [102]. However, DADS eliminated the toxic effect of trans-crotonaldehyde by interaction with its –C=C–C– and –CH=O groups [103].

### 3.6. Neuroprotection

Garlic and garlic extracts are believed to provide therapeutic benefits in neurological disorders owing to their antioxidant, anti-inflammatory, and neuroprotective effects [3, 104]. A recent study found that DADS (40 or 80 mg/kg) effectively improved LPS-induced depression-like behaviours in mice, with treatment effects comparable to those of imipramine (10 mg/kg), a clinical antidepressant [105]. However, in young mice, especially during the neural growth stages, high doses of DADS may adversely affect hippocampal neurogenesis, the proliferation of neural progenitor cells, and neurocognitive functions by regulating ERK and brain-derived neurotrophic factor (BDNF)/cAMP response element-binding protein (CREB) signaling, resulting in significant memory deficits [106]. Besides, another recent animal study has shown that DADS played a role in the inhibition of neuropathic pain via the H_2_S/BDNF/Nrf2 pathway [107].

Several previous studies have suggested that DADS may be an effective drug for the treatment of neurodegenerative disorders, such as Alzheimer's disease (AD). Animal studies have shown that DADS could ameliorate the learning and memory of AD mouse models by increasing the number of hippocampal dendritic spines and synapses [108]. DADS derivatives, 7k and 7l, inhibited A*β*-induced neuronal cell death and reverse scopolamine-induced cognitive impairment in rats via their antioxidative and metal-chelating effects [109, 110]. Moreover, DADS exerted antiamyloidogenic and anti-inflammatory effects and inhibited conformational alteration in tau protein induced by phosphorylation via the GSK-3*β* pathway [111]. A clinical trial found that the severity of some neurodegenerative diseases, such as AD, was associated with H_2_S levels. Therefore, as DADS is an H_2_S donor; it may play a role in the treatment of AD [112].

### 3.7. Anticancer Activity

#### 3.7.1. Inhibition of Invasion and Migration

The inhibitory effect of DADS on cancer cell movement and invasiveness is identified to be linked to the enhancement of tight junctions and the decrease in MMPs activity [113, 114]. Increases in transepithelial electrical resistance confirmed that DADS enhances the tight junctions of human prostate cancer cells [113]. DADS was found to block the migration and invasion of human colon cancer 205 cells by inhibiting the expression of MMP-9, MMP-2, and MMP-7 [115]. Additional evaluations revealed that the effect of DADS on MMPs was regulated through the NF-*κ*B and PI3K/Akt pathways [116]. Previous studies had shown that DADS could reduce TNF-*α*-induced C–C motif chemokine ligand 2 release, thereby blocking monocyte recruitment and inhibiting malignant tumor invasion [117, 118].

The prevention of epithelial-mesenchymal transition (EMT) is a new hotspot in tumor metastasis research. Inhibiting Ras-related C3 botulinum toxin substrate (Rac)-1 and *β*-catenin expression can inhibit EMT in tumor cells [119]. According to studies by Su et al. [120], DADS suppressed the activities of Rac1, *β*-catenin, p21 activated kinase-1, and Rho kinase-1, leading to the inhibition of gastric tumor cell growth, invasion, and metastasis. Furthermore, DADS regulated MMP-9 expression and reversed EMT by inhibiting the *β*-catenin pathway to reduce breast cancer cell metastasis [121]. Inhibition of the LIMK1-cofilin1 pathway by DADS also inhibited EMT, migration, and invasion of gastric cancer cells, which are closely associated with the formation of invasive pseudopods [122]. Notably, these findings were also confirmed using colon cancer cells [123, 124]. Fibronectin, an extracellular matrix component, also causes EMT in tumors. However, treatment with DADS has been reported to reverse the EMT induced by fibronectin in tumors [125]. The deglycase-1 (DJ-1) protein is another promising target for cancer therapy owing to its roles in invasion, migration, and chemoresistance, and several reports have suggested that inhibition of Src phosphorylation by DADS could downregulate DJ-1 expression, thereby inhibiting leukemic cell migration and invasion [126].

#### 3.7.2. Regulation of Cell-Cycle Arrest

DADS was found to inhibit the proliferation of tumor cells partly because of its ability to reduce the cell ratio in the G1 phase and increase the cell ratio in the G2/M phase [127]. During treatment with DADS, the proportion of G2/M cells increased with increasing concentration and exposure time. Further molecular analysis indicated that the reduced level of cyclin B1, cell division cycle (cdc) 25C, cdc2, and phosphorylated-cdc2 proteins may have contributed to the blockage of the G2/M phase in DADS-treated esophageal squamous cell carcinoma cells [128]. Studies have shown that DADS increased the mRNA and protein levels of p21 and p53 in carcinoma cells and activated the p53/p21 signaling pathway, thereby inducing cell-cycle arrest and cell apoptosis [128, 129]. A previous study indicated that the ability of DADS to block the cell cycle was also associated with histone acetylation [130]. Further research demonstrated that DADS induced an increase in histone H3 and H4 acetylation in the CDKN1A promoter, ultimately leading to an increase in CDKN1A gene expression and p21^WAF1^ protein levels [131]. Moreover, DADS resisted the activation of the G2/M gene damage checkpoints by relying on Mec1 (ATR) and Tel1 (ATM) to inhibit DNA repair, which could improve the efficacy of DNA damage-based cancer therapies [132].

Some garlic extracts, including DADS, exert antimitotic effects by impairing microtubules and hindering the assembly of mitotic spindles. Aquilano et al. [133] reported the obvious loss of the microtubule network, with an irregular accumulation of soluble *β*-tubulin and reduction of the cytoskeletal counterpart in neuroblastoma SH-SY5Y treated with DADS. In addition, DADS-derived superoxide was observed to actively participate in the oxidation of actin and tubulin, which eventually led to the breaking of the microfilaments and microtubules.

#### 3.7.3. Induction of Apoptosis and Autophagy

Inducing apoptosis in cancer cells is the main anticancer mechanism employed by most chemotherapeutic drugs [134]. DADS-induced apoptosis was observed to be accompanied by an increase in Ca^2+^ levels and a decrease in mitochondrial membrane potential. Increased Ca^2+^ led to the activation of caspase-3 and the release of cytochrome C from the mitochondria, resulting in proteolysis and apoptosis [135]. In addition to caspase-3, caspase-9 and caspase-10 were also activated by DADS [136]. Exposure to DADS increased the expression of p53, p38, and p21; decreased the level of antiapoptotic protein, Bcl-2; and upregulated the levels of the proapoptotic proteins, Bax and Bad [127, 137–139]. Moreover, inhibition of histone deacetylation and the ERK pathway and activation of the SAPK/JNK pathway were also found to influence the proapoptotic effect of DADS in human breast cancer [140]. Several studies have also revealed that treatment with DADS could lead to an increase in ROS levels, resulting in the apoptosis of human leukemia HL-60 cells [141, 142]. However, cells with an ROS buffer system, such as adenocarcinoma gastric cells (rich in glutathione peroxidase) or copper-overexpressing neuroblastoma cells, were shown to be resistant to DADS treatment [143, 144]. One animal experiment showed that pretreatment with 10 *μ*M DADS resulted in an increase in the radiation sensitivity of HeLa cells and significantly promoted radiation-induced apoptosis. Such findings indicated that DADS is a potential radiosensitive agent for human cervical cancer [145].

In addition to inducing apoptosis, some chemotherapeutic drugs induce autophagy, which is another cell death pathway. Studies have reported that exposure to DADS significantly increased the autophagic flux of RAW264.7 cells, and the effects of DADS on autophagy were likely the result of inhibition of the phosphorylation of mTOR and P70S6k/S6K1 [146]. DADS-induced autophagy increases the death of tumor cells, including leukemia and osteosarcoma cells, by inhibiting the PI3K/Akt/mTOR signaling [147–149]. It has been suggested that histone deacetylase (HDAC) inhibitors also play an antitumor role through autophagy [150]; thus, the inhibitory effect of DADS on HDAC activity may partially induce autophagy. However, there is a paucity of research in the field of DADS-induced autophagy, and more investigations are warranted.

#### 3.7.4. Induction of Cell Differentiation

DADS-induced differentiation of human leukemia HL-60 cells was found to be related to the decrease in DJ-1 and calreticulin (CRT) contents [151]. DJ-1 has been reported to play a role in cell differentiation by acting as a cofactor-binding protein or transcription factor [152]. DADS significantly decreased the expression of cluster of differentiation 33 (CD33) and increased the expression of CD11b by downregulating CRT, ultimately inducing the differentiation of human leukemia HL-60 cells [153]. Furthermore, the DADS-induced reduction of CRT could upregulate the mRNA expression of CCAAT enhancer-binding protein-*α*, thereby affecting cell differentiation [154]. Moreover, treatment with DADS was found to increase the acetylation level of core nucleosome histones (H3 and H4) and accelerate the differentiation of human leukemia cells [155, 156] and liver cancer cells [157].

#### 3.7.5. Effect on Epigenetics

The blocking of normal histone acetylation or abnormal histone acetylation is believed to be the root cause of several cancers. DADS was found to enhance the acetylation of histones H3 and H4 in normal colon cells both *in vitro* and *in vivo* [158]. Druesne et al. [159] reported that treatment with DADS alone increased the transient acetylation of histone H3K14 in human colon tumor cells. However, unlike in normal colon cells, DADS had no effect on histone H4 acetylation in colon tumor cells, regardless of the cell culture conditions. Furthermore, DADS induced an increase in histone acetylation of the CDKN1A promoter, which in turn led to an increased level of the p21^WAF1^ protein; this process is known to inhibit tumor proliferation and induce G2/M phase arrest and apoptosis [160]. Notably, these effects of DADS were only observed at high concentrations. Further research is thus needed to confirm whether the HDAC inhibitory effect of DADS can result in primary anticancer effects when normal human diet doses are administered.

### 3.8. Regulation of Metabolism

#### 3.8.1. Regulation of Glycose Metabolism

Several *in vivo* studies have shown a dose-dependent increase in blood glucose concentration and free fatty acid levels in rats treated with DADS. Such findings suggest that DADS affects glucose metabolism [161]. However, another study reported that garlic oil, rather than DADS, had beneficial effects on glycemic control in streptozotocin-induced diabetic rats [162]. As a result, the specific effects of DADS on glucose metabolism, under both healthy and diabetic conditions, need to be further elucidated. In addition, DADS was observed to suppress glucose metabolism of breast cancer stem cells by inhibiting the CD44/pyruvate kinase M2/AMPK pathway [163].

#### 3.8.2. Regulation of Lipid Metabolism

According to reports, DADS may regulate lipid metabolism by: (a) regulating sterol regulatory element-binding protein-1c, apolipoprotein A1, CREB-H, and fibroblast growth factor 21; (b) preventing lipotoxicity by increasing peroxisome proliferator-activated receptor-*α* and inhibiting stearyl coenzyme A desaturase enzyme-1; and (c) significantly inhibiting lipid peroxidation by regulating malondialdehyde and superoxide dismutase [164–166]. Additional studies have reported that the lipid metabolism-regulating activity of DADS may have significant hepatoprotective effects [3]. Additionally, DADS could inhibit the accumulation or activation of mesenteric adipose tissue macrophages and the release of monocyte chemoattractant protein-1, suppressing the inflammatory response induced by obesity [167].

### 3.9. Other Effects

Oral administration of DADS increased the activity of the natural antibody in broiler serum [168]. Moreover, DADS induced chromosome aberration and sister chromatid exchange in the Chinese hamster ovary [169]. DADS could also change iron homeostasis by regulating the expression of ferritin and transferrin receptor genes in hepatocytes *in vitro* and *in vivo* [170] (see Figure 2).

## 4. Conclusions and Prospects

DADS, a natural organic sulfur compound, is commonly used as a food additive. Current research suggests that DADS is a promising drug agent for the prevention and treatment of several diseases. This review sought to systematically identify the biological functions of DADS and summarize the underlying molecular mechanisms employed by this compound. The biological functions of DADS can be divided into two categories: the protective effects on normal tissues and the inhibitory effect on disease status. The anti-inflammatory and antioxidant effects of DADS are the basis for maintaining tissue homeostasis (such as neurovascular protection and metabolic regulation) and fighting infections (antibiosis). There are interlinks between the anti-inflammatory and antioxidant effects, with NF-*κ*B and ROS signaling playing key roles. DADS alters the biological properties of cancer cells via specific intracellular and intercellular mechanisms. As a result, DADS exerts significant anticancer effects, such as inducing apoptosis, autophagy, and differentiation. In addition, DADS can also improve efficacy and reduce the negative effects of chemotherapy drugs.

Anti-inflammatory and antioxidant signaling mediators, such as NF-*κ*B, TNF-*α*, ROS, Nrf2, AP-1, JNK, and STAT, play important roles in the biological functions of DADS. Apoptosis and autophagy-associated pathways, such as PI3K, Akt, mTOR, MAPKs, Bcl-2, and Bax, also contribute to the anticancer action of DADS. Notably, the signaling pathways affected by DADS are similar between normal tissue cells and cancer cells. However, different dosages and methods of administration may produce different effects, which requires more experiments to fully verify (see Figure 3).

There are some clinical trials focusing on garlic and its biological effects, including anticancer, anti-inflammatory, antioxidant, and antiviral activities [64, 171–173]. These clinical studies have shown that garlic can be used as an adjunct in the management of several diseases, but with limited effects. Further clinical trials on solitary compounds are necessary to identify the specific active ingredients and thus enhance their medicinal value. Although animal and *in vitro* experiments have shown that DADS has comparable biological activity with garlic, clinical trials of DADS have not yet been conducted. Therefore, it is still unclear whether DADS is an active ingredient in the use of garlic in humans and how it exerts its effect. It should be noted that there are some non-negligible issues that need to be solved before conducting clinical trials of DADS. The first is that DADS is rapidly metabolized after being taken into the body and has low bioavailability [6]. The second is the technical difficulties of processing DADS, such as characterization, optimization, and the production of suitable delivery systems [174, 175]. The most important issue is the pharmacokinetic studies of DADS, and its metabolites should be refined. Currently, countries are probing different strategies to prevent and treat COVID-19, which has had a negative impact on global public health and economies. Readily available natural plant products could be a promising starting point for the discovery of new therapeutic drugs. Research on the biological function of DADS may bring us new hope.

## Figures and Tables

**Figure 1:** Chemical structure of DADS.

**Figure 2:** Overview of the biological functions of DADS.

**Figure 3:** The signaling pathways affected by DADS.
